This article has been retracted.

# Barriers and facilitators of childhood obesity prevention policies: A systematic review and meta-synthesis

**DOI:** 10.3389/fped.2022.1054133

**Published:** 2023-01-11

**Authors:** Shahnaz Taghizadeh, Mohamad Ghazanfari Hashemi, Rahim Khodayari Zarnag, Ehsan Fayyazishishavan, Marjan Gholami, Mahdieh Abbasalizad Farhangi, Leila Jahanbazi Gojani

**Affiliations:** ^1^ Department of Community Nutrition, Faculty of Nutrition, Tabriz University of Medical Sciences, Tabriz, Iran; ^2^ School of Medicine, Tehran University of Medical Sciences, Tehran, Iran; ^3^ Department of Health Policy and Management, School of Management and Medical Informatics, Tabriz University of Medical Sciences, Tabriz, Iran; ^4^ Department of Biostatistics and Data Science, School of Public Health, The University of Texas Health Science Center at Houston (UTHealth), Houston, TX, United States; ^5^ Department of Pharmacy, Faculty of Pharmacy, Islamic Azad University Pharmaceutical Sciences Branch, Tehran, Iran; ^6^ Drug Applied Research Center, Tabriz University of Medical Sciences, Tabriz, Iran; ^7^ Student Research Committee, Tabriz University of Medical Sciences, Tabriz, Iran

**Keywords:** barriers, facilitators, childhood obesity, prevention, policies barriers, policies

## Abstract

**Objectives:**

Childhood obesity is one of the worldwide considerable public health challenges and many factors can play a role in its management. Therefore, this article examined the facilitators and barriers of childhood obesity prevention (COP) policies.

**Methods:**

This systematic review of qualitative studies was conducted *via* a search of the SCOPUS, PubMed, and Google Scholar databases between 1 January 2010 and 11 February 2022 and examined factors that influence the implementation of COP policies at a community approach.

**Results:**

The parents' reluctance to engage in COP activities, lack of sufficient knowledge, and financial problems were the most reported barriers at the individual level. In addition, the beliefs about COP at the sociocultural level and limited funding and resources, time limitations in stakeholders at the implementation level, and lack of policy support at the structural level were the most frequently reported barriers. Further, effective communication between stakeholders and parents and school staff at the sociocultural level and flexibility of the intervention, delivery of healthy food programs in schools, low-cost and appropriate resources, and the availability of appropriate facilities are the most frequently reported facilitators in the structural level.

**Conclusion:**

Individual, sociocultural, and structural level-related barriers and facilitators influence the implementation of COP policies. Most of the barriers and facilitators in this systematic review were related to the structural level.

## Introduction

Childhood obesity is a considerable public health challenge with numerous health, economic, and social consequences. Nearly one in five children and adolescents is overweight or obese (1). The complications and problems of childhood have been widely demonstrated (2–4). Children with obesity are at a greater risk of obesity in adulthood; a recent study showed that 70% of adolescents with obesity remained obese at the age of 30 years (5). In 2015, studies showed that overweight and obesity accounted for about 4 million deaths worldwide, and almost 70% of these deaths were due to cardiovascular disease. Other chronic outcomes of obesity in addition to cardiovascular disease include pre-diabetes and diabetes mellitus, increased risk of severe musculoskeletal diseases, and many others (6–9). The incidence of cardiometabolic diseases in adolescents with obesity is significantly higher than in adolescents of normal weight (10). Most of the studies reported an increase in the prevalence of childhood obesity at a high rate (11, 12), while some others reported this prevalence at a slower rate (13–15). Numerous factors have been attributed to affect the prevalence of childhood obesity. The Ecological Model of Growth (EMG) in childhood, as a combination of Bronfenbrenner's ecological theory (16, 17) and Reifsnider's epidemiology models (18), suggests that the levels of individual characteristics (e.g., gender, age, and preference), microsystem (e.g., family, teachers, and friends), mesosystem (e.g., neighborhood, school, and physical family), and exosystem (e.g., economics, culture, and politics) contribute to the development of childhood obesity (19). Various interventions have been performed to prevent obesity in this age group (20–24); however, the effectiveness of these interventions was confirmed in some of the communities (20, 23, 24) but not others (21, 22). Regarding the multidimensional nature of childhood obesity (25), studies suggested that effective interventions in the prevention of childhood obesity require the participation of stakeholders and organizations at various levels and sectors (26) with a coordination of cross-sectorial partnerships (27), not only at small-scale levels, such as schools or families, but also at the large-scale levels of community with particular supports of multiple sectors and environments (28). Studies also demonstrated that lack of funding and the extent of temporary disruptions in long-lasting interventions impairs the long-term efficacy of childhood obesity prevention (COP) policies (29). According to the report by Adab et al., reducing the proportion of children with excess weight is an important characteristic of effective COP policies (28). Therefore, an investigation of the barriers and facilitators of the COP policies is one of the necessary requirements of this field.

To the best of our knowledge, no study systematically examines the barriers and facilitators of COP policies, and existing studies are usually limited to specific settings or topics, such as school-based interventions, or a focus on physical activity (30–32), healthy eating (33–35), or the perspectives of adolescents on these issues (36). Therefore, the aim of the present study was to conduct a comprehensive review of the barriers and facilitators of COP policies.

## Materials and methods

The current systematic review was prepared according to the Preferred Reporting Items for Systematic Reviews and Meta-Analyses (PRISMA) statement (37). The study protocol was registered in the International Prospective Register of Systematic Reviews (PROSPERO) system (Identifier: CRD42019138359) and has also been approved by the ethics committee of Tabriz University of Medical Sciences (registration no. IR.TBZMED.VCR.REC.1400.572).

### Data source and search strategy

The search for resources was conducted in SCOPUS, PubMed, and Google Scholar. Search terms (policy, program, pediatric obesity, childhood obesity, prevention, facilitators, driving force, barriers, inhibitors) were comparable between databases. All articles were considered eligible when they were qualitative studies and published between 1 January 2010 and 11 February 2022, which examined factors that influence the implementation of COP policies at a community approach. No language restriction was applied.

A sample search strategy in PubMed is presented in Supplementary Table S1. We reviewed the reference lists of all related and available articles to prevent missing any information. The selection criteria of this review were independently identified by two researchers.

### Eligibility criteria and study selection

All articles that examined factors that influenced the implementation of COP policies in a community approach were considered eligible. These factors could impede, prevent, or facilitate the implementation of COP policies. For this review, a barrier was defined as an obstacle or circumstance that keeps things or people apart or prevents communication or progress, or any factor (e.g., person, place, context, or emotional state) that restricts the implementation of comprehensive obesity prevention interventions in children and adolescents, whereas a facilitator was defined as a thing or person that makes something possible and applicable (38, 39).

### Quality assessment and data extraction

The risk of bias and study quality were assessed using the Critical Appraisal Skills Program (CASP) checklist for the reporting of all qualitative studies (40, 41), which contains 10 questions. The quality of the studies was evaluated by two researchers. After carefully studying the full text of each article, the quality evaluation checklist was completed by the first researcher and the items were scored. The same method was re-evaluated by the second researcher. Since there were 10 attributes (questions), and the maximum score for each attribute was 5, the maximum score that each article received based on the CASP scale was 50. According to the previous report (42), the studies that were scored as 75% or more of the maximum attainable score (≥37.5 points) were considered to be “high-quality” studies. Studies that were scored 50%–75% (25–37.5 points) were considered to be “moderate-quality” studies, and studies with scores below 50% (≤25 points) were considered to be “low-quality” studies. General study characteristics (e.g., author, year of publication, country, the aim of the study, sample size, participants, data source, place of study, statistical analysis, and quality of study) were extracted from included studies.

### Data synthesis

Barriers and facilitators that were reported in the studies were synthesized using the Theoretical Domains Framework (TDF) (43). The TDF framework is recommended to identify the barriers and facilitators of the implementation of COP policies and has been applied in community-based studies (44–46). By summarizing the domains in this framework, we identified three main themes: individual, sociocultural, and structural factors. Two authors separately coded the barriers and facilitators based on the definitions of Cane et al. (43). Any disagreements were resolved by a review from a third author.

## Results

### Study selection

A search of the electronic databases retrieved 6,679 records; after removing duplicates, 6,468 articles were screened by title and abstract (Figure 1). The remaining 400 full-text articles were screened, and 22 publications were included in the qualitative synthesis. A gray literature search did not identify any published results for policies in this scope.

**Figure 1:** Flow chart of study selection.

### Study characteristics

The study and participant characteristics are presented in Table 1. This review draws on the findings of 22 studies with a total of 1,039 participants. Studies have been performed on different settings of healthcare centers (*n* = 5) (48, 50, 55, 56, 60), schools (*n* = 8) (39, 49, 51, 53, 54, 57, 58, 64), stakeholders offices (*n* = 4) (47, 59, 61, 66), school and stakeholders offices (*n* = 2) (65, 67), and two studies were conducted online (52, 63). The identified papers reported research conducted in 12 countries: the United States (*n* = 6) (55, 61, 63, 64, 66, 67), South Korea (*n* = 1) (48), the United Kingdom (*n* = 2) (49, 57), Sweden (*n* = 1) (50), Ireland (*n* = 1)(51), Malaysia (*n* = 2) (47, 52), Brunei (*n* = 1) (53), Columbia (*n* = 1) (54), Australia (*n* = 2) (56, 60), Saudi Arabia (*n* = 1) (39), the Netherlands (*n* = 1) (58, 59), Africa (*n* = 1) (62), and Canada (65). Three studies were a combination of focus groups and interviews (48, 49, 66), fifteen studies were interviews (39, 47, 50, 51, 53–55, 57–59, 61, 62, 64, 65, 67), two studies used online questionnaires (52, 63), one study used nominal group technique (56), and one study used focus group discussions (60). The quality of the studies was evaluated by two researchers and the kappa coefficient showed the agreement between the two researchers. The quality of studies was moderate for 11 studies (49, 50, 53–55, 57, 58, 63, 64, 66, 67) and high for 11 studies (39, 47, 48, 51, 52, 56, 59–62, 65) (Table 2).

**Table 1:** Characteristics of included studies.

First author, year (reference)	Country	Aim of study	Sample size	Participants	Data source	Setting	Analysis	Quality^a^
Almutairi, 2022 (39)	Saudi Arabia	The perception of school principals and sports teachers about barriers and enablers to implementing obesity prevention strategies	14	School principals and sports teachers	Interviews	School	Thematic analysis	High
Ng, 2021 (47)	Malaysia	Investigate the policy processes relating to food marketing to children in Malaysia	9	Federal government, food industry, and civil society stakeholders	Interviews	Stakeholders offices	Thematic analysis	High
Park, 2020 (48)	South Korea	Service providers’ perspectives on barriers to improving healthy eating	18	Service providers and assistant cooks at community childcare (CCC) centers	Focus group and interviews	CCC centers	Thematic analysis	High
Malden, 2020 (49)	UK	Assessing the acceptability of ToyBox intervention	13	Parents and teachers	Focus groups and interviews	School	Thematic analysis	Moderate
Sjunnestrand, 2019 (50)	Sweden	Child health care nurses’ perceptions about overweight and obesity	17	Child health care (CHC) nurses	Interviews	CHC centers	Thematic analysis	Moderate
Hayes, 2019 (51)	Ireland	Barriers and facilitators to obesity prevention interventions	15	Key stakeholders	Interviews	School	Thematic analysis	High
Chan, 2018 (52)	Malaysia	Facilitators and barriers obesity prevention for primary school children	447	School administrators	Online questionnaire	Online	Logistic regression	High
Ahmad, 2018 (53)	Brunei	Barriers to effectively addressing the issue of childhood obesity	17	Health and education government agencies and school community members	Interviews	School	Thematic analysis	Moderate
Schroeder, 2017 (54)	Columbia	Barriers and facilitators of school nurses experience in implementing obesity intervention	19	School nurses	Interviews	School	Content analysis and heat mapping	Moderate
Dev, 2017 (55)	USA	Childcare providers’ perspectives about nutrition education for children	18	Childcare providers	Interviews	Childcare centers	Thematic analysis	Moderate
Cyril, 2017 (56)	Australia	Barriers and facilitators to childhood obesity prevention	29	Parents	Nominal group technique	Health service setting	Software Stata (only has descriptive data)	High
Clarke, 2017 (57)	UK	Head teacher perspectives of obesity prevention in primary schools	22	Head teacher	Interviews	School	Thematic analysis	Moderate
Van, 2016 (58)	Netherlands	Barriers and opportunities for Dutch obesity Intervention in teenagers (DOiT)	44	Teachers and Dutch Obesity Intervention in Teenagers (DOiT) coordinators	Interviews	School	Thematic analysis	Moderate
Hendriks, 2016 (59)	Netherlands	Obstacles and enablers on the way toward Integrated physical activity policies for childhood obesity prevention	15	Policy officials from health and nonhealth policy domains	Interviews	Stakeholders offices	Framework approach to deductively analyze	High
Cyril, 2016 (60)	Australia	Service providers’ perspectives in improving childhood obesity prevention	59	Service providers	Focus group discussions	Health service setting	Thematic analysis	High
Chuang, 2016 (61)	USA	Factors affecting implementation of the childhood obesity program	74	Leaders and key stakeholders	Interviews	Offices	Thematic analysis	High
Phillips, 2016 (62)	Africa	Perceptions of diet, physical activity, and obesity-related health	32	Daughter–mother pairs	Interviews	Hospital	Thematic analysis	High
Totura, 2015 (63)	USA	Assessing implementation of childhood obesity prevention strategies in schools	62	School health professionals	Online questionnaire	Online	Multiple regression and slope analyses	Moderate
Fagen, 2014 (64)	USA	Opportunities and challenges in school-based obesity prevention	25	School district personnel	Interviews	School	Qualitative data analysis software (ATLAS)	Moderate
Mâsse, 2013 (65)	Canada	Implementation of physical activity and food policies in schools	50	Principals and key teachers/school informants	Interviews	School and stakeholders offices	Thematic analysis	High
Trudnak, 2012 (66)	USA	The childhood obesity response	26	Stakeholders from private and public organizations	Focus groups and interviews	Department of Health and Education	Thematic analysis	Moderate
Patel, 2012 (67)	USA	Barriers to the implementation of obesity prevention policies in elementary schools	14	Stakeholders at the district- and school-levels	Interviews	The district and school	Empirical analysis	Moderate

^a^ The quality of the studies were assessed using the Critical Appraisal Skills Program (CASP) checklist.

**Table 2:** The Critical Appraisal Skills Program (CASP) checklist for quality assessment of studies.

Study Question	(39)	(47)	(48)	(49)	(50)	(51)	(52)	(53)	(54)	(55)	(56)	(57)	(58)	(59)	(60)	(61)	(62)	(63)	(64)	(65)	(66)	(67)
Q1	5	5	5	5	4	5	5	5	5	5	5	5	2	5	5	0	5	3	5	4	5	3
Q2	4	5	4	2	3	4	4	3	3	3	3	3	4	5	5	4	3	4	3	4	3	3
Q3	5	4	4	4	3	5	5	4	4	3	4	3	3	5	5	5	4	3	4	5	3	4
Q4	4	3	4	4	5	5	5	3	4	3	5	3	4	4	5	5	5	3	4	5	4	4
Q5	5	5	5	4	3	5	5	3	4	4	4	3	5	5	5	5	4	4	4	4	4	4
Q6	5	4	4	4	2	3	4	3	3	3	4	3	3	4	4	5	5	2	3	4	5	4
Q7	5	5	1	2	5	5	5	5	1	1	5	5	2	5	5	1	5	2	2	4	1	2
Q8	5	5	5	4	4	4	5	4	4	4	3	4	4	5	5	5	4	5	4	5	4	4
Q9	5	4	4	5	3	3	5	4	3	4	5	3	5	5	4	5	3	4	3	5	3	3
Q10	5	4	5	3	4	5	5	3	5	4	5	4	5	5	5	5	3	4	5	5	5	5
Total Score	**48**	**40**	**41**	**37**	**36**	**44**	**48**	**37**	**36**	**34**	**43**	**36**	**37**	**48**	**48**	**40**	**41**	**34**	**37**	**45**	**37**	**36**
Quality Status	**H**	**H**	**H**	**M**	**M**	**H**	**H**	**M**	**M**	**M**	**H**	**M**	**M**	**H**	**H**	**H**	**H**	**M**	**M**	**H**	**M**	**M**

Q1: Was there a clear statement of the aims of the research? Q2: Is a qualitative methodology appropriate? Q3: Was the research design appropriate to address the aims of the research? Q4: Was the recruitment strategy appropriate to the aims of the research? Q5: Was the data collected in a way that addressed the research issue? Q6: Has the relationship between researcher participants been adequately considered? Q7: Have ethical issues been taken into consideration? Q8: Was the data analysis sufficiently rigorous? Q9: Is there a clear statement of findings? Q10: How valuable is the research?

H, high quality; M, moderate quality.

### Analysis of included studies

A total of 60 barriers (Table 3) and 27 facilitators (Table 4) emerged from the thematic analysis. Barriers and facilitators were categorized into three main categories.

• Individual level: These factors included items in which the stakeholders either benefit from the policies or the stakeholders are only policy implementers without involvement and role in policymaking. A total of 17 barriers were reported in the individual factors.
• Sociocultural level: These factors included in the policy are those that are beyond the individual level and items that are widespread in the context of the society or have origins in the culture of that society and are not related to the policymaking or policy implementers. Eight barriers and 13 facilitators were reported in the sociocultural factors.
• Structural level: Finally, structural factors express the items that are related to the different dimensions of decision making and policymaking. In total, 35 barriers and 14 facilitators were reported in the sociocultural factors.

**Table 3:** Barriers of childhood obesity prevention policies

Themes	Barrier (reference)
Individual level (*N* = 17)	Lack of risk perception in children (48) Lack of Self-regulation and self-control when eating in children (48) Lack of coping skills in children (48) lack of access to sports teams (62) feeling tired in the children (62) Lack of confidence in CHC nurses communication skills (50) Lack of sufficient knowledge in nurses (50) Lack of sufficient knowledge in parents (56, 60) Difficulties in health information utilization among parents (60) Low parent participation rates (67) Poor utilization of maternal and child health services by parents (60) Lack a sense of responsibility in assistant cooks (48) Little or no knowledge in assistant cooks (48) Lack of active transport by parents (51) Parents’ financial problems (48, 62) Parent's reluctance to become involved in COP activities (51, 53, 67) Language problem (56)^a^
Sociocultural level (*N* = 8)	Insufficient cooperation with other healthcare providers in nurses (50) Cycling is unsuitable for girls (51) Cycling to school is unsafe (51) Nurses concerns about discuss of obesity stigma as a barrier to the parents (60) Cultural beliefs on childhood obesity (56, 60, 66) Teamwork (59) Passive managerial commitment (59) Existence of misinformation in the society (66)
Structural level (*N* = 35)	Lack of space in the building (49, 57) Time limitations in stakeholders in the implementation level (49, 51, 52, 60, 62, 66) Program accessibility barriers in parents (56) Top-down process (59) Lack of monitoring (47) Insufficient cooperation with other healthcare providers in nurses (50) Conflicting policies within preschools (49) Problems in agenda setting (59) Insufficient training (52, 63) Lack of clear childhood obesity and policies effectiveness data (51, 60) Lack of infrastructure near schools (39, 51) Absence of a travel plan (51) Lack of equipment and facilities (52, 53) insufficient workforce (53) Competing priorities^b^ (53, 65) Parents and administrative principals as preventing the implementation of interventions (54) Obesogenic environments (54) Limited funding and resources at the executive level (47, 55, 61, 63–67) Restrictive policies (55) Junk food advertisement (47, 56) Lack of mandatory weight checks for schoolchildren (56) Academic pressure (57) Lack of external, institutional and experts support of policy (53, 57, 63, 65–67) Lack of planning (58) Other urgent unforeseen priorities (58) No plan to cope with teacher and staff turnover (58, 61, 64) High teacher or nurse workload (54, 58) Operational level policy formulation (59)^c^ Inadequate dietetic services (60) Limited local control over food provided in schools (39, 61) Lack of strategy and policy guidelines clarity (47, 60, 63) Lack of buy-in (64) Legal roadblocks (64) Magnitude of the obesity problem (66)

^a^ Language problem: The community language is other than language at home.

^b^ Competing curriculum demands and priorities or competing commitments/priorities in the schools.

^c^ Formulation appropriate policies and not implement them properly at the operational level.

**Table 4:** Facilitators to childhood obesity prevention policies.

Themes	Facilitator (reference)
Sociocultural level (*N* = 13)	User-friendliness of the intervention materials (49) Staff members (52) Commitment of schools staffs, canteen operators and students (52) Good relationships and teamwork with parents and school staff (54, 57) Bicultural playgroup leaders (54, 56) Ethnic community groups (56) Strong teacher motivation (58) Taking a participatory approach to the development of program materials (61) School districts with existing collaborations (39, 64) Effective communication between stakeholders (58, 64, 67) Obesity messages for the public (66) Obesity messages for policymakers (66) Obesity messages for clients (66)
Structural level (*N* = 14)	Integration of the intervention with the curriculum (49) Flexibility of the intervention (49, 58) Delivery of healthy food program in schools (39, 51, 56) Involvement of the police in traffic workshops in the school (51) Access to feasible resources (47, 55) Low-cost and appropriate resources (55, 65) Work around restrictive policies to accommodate nutrition education (55) Use of experts from external agencies (57) The availability of appropriate facilities (57, 65) Involvement of intervention providers’ coordinator (58) Gradually introducing activities (61) Minimizing staff burden (61) Formal and informal leaders (47, 64) Appropriate support of intervention (58, 65)

#### The individual-level barriers

The most frequently reported and important barriers in the individual level were parents' reluctance to become involved in COP activities (51, 53, 67), lack of sufficient knowledge (56, 60), and financial problems (48, 62). The other individual-level barriers related to parents (51, 60, 67), children themselves (48, 56, 62), nurses (50), and assistant cooks (48) are shown in Table 3.

#### The sociocultural-level barriers

The most frequently reported and important barriers in the sociocultural level were cultural beliefs on childhood obesity (56, 60, 66). The other barriers in this level include concerns about obesity stigma (60), the barriers related to executive managers (50, 59), social security about cycling (51), and cycling being unsuitable for girls (51).

#### The structural-level barriers

Most of the barriers in this systematic review were related to the structural level, of which 32 barriers were extracted. The most important and frequently reported barriers at the structural level were limited funding and resources (47, 55, 61, 63–67), time limitations of the stakeholders in the implementation level (51, 52, 60, 62, 66), and the lack of external, institutional, and experts’ support of the program (53, 57, 63, 65–67). The other structural-level barriers (49, 51–61, 63–66) with their details are shown in Table 3.

The facilitators of the COP policies in this study are shown in Table 4. The facilitators were at the sociocultural and structural levels, and no facilitator at the individual level was identified in the studies included in this review.

#### The sociocultural-level facilitators

The most frequently reported sociocultural-level facilitators were effective communication between stakeholders (58, 64, 67), and good relationships and teamwork with parents and school staff (54, 57). Other student and school staff-related facilitators (52, 58, 61, 64) as well as facilitators related to parents (56) and obesity messages for the public, policymakers, and clients (66) are shown in Table 4. Trudnak et al. suggested that messages for clients should be simple and direct, such as the 5-2-1-almost none, for policymakers should be “backed by data,” “direct,” and solutions-oriented and, for the public, include social marketing campaigns (66).

#### The structural-level facilitators

The flexibility of the intervention (49, 58), delivery of healthy food programs in schools (39, 51, 56), low-cost and appropriate resources (55, 65), and the availability of appropriate facilities (57, 65) are the most frequently reported facilitators in the structural level. Other structural-level facilitators (49, 51, 52, 55, 57, 58, 61, 64, 65) are shown in Table 4.

## Discussion and conclusion

The aim of the present study was to describe barriers and facilitators that may influence the implementation of COP policies. The review found that individual-, sociocultural-, and structural-level barriers and facilitators have the greatest effect on COP policies; however, most of the barriers and facilitators in this systematic review were related to the structural level.

The results of this review should be discussed considering its limitations and strengths. To our knowledge, this is the first comprehensive review that synthesizes the barriers and facilitators of COP policies in all of the possible dimensions, in different settings, and all societies. Several limitations of this research must be acknowledged. First, due to the nature of the study, certain stakeholders must be interviewed that may stem for selection bias. However, this selection was necessary because there were specific stakeholders in each of the organizations who were interested in the COP policies. Second, mixed-method studies pay less attention to the results of qualitative investigations and focus more on quantitative results. This indicates that future research in this field should seek to address these risks to ensure certain factors such as culture, service location, and socioeconomic status are adequately captured. Third, there was a lack of information on individual facilitators and this case of facilitators was ignored by most of the studies. Across the 22 included studies, three relatively important barriers to COP policies emerged: the most important barriers at the individual level were related to the parents, which include parents’ reluctance involves of policies (51, 53, 67), insufficient knowledge (56, 60), and financial problems (48, 62). These results are consistent with the study by Ray et al. (68), which suggested that when parents themselves raised concerns about their child's weight, they were more likely to engage in COP policies (68). Financial problems in the family mean that parents may spend more time on work, with less capacity to participate in the intervention policies (66, 69). Insufficient knowledge and program accessibility barriers may exacerbate this situation. Paes et al. demonstrated that negative parental patterns in purchasing inappropriate foods, preference for buying, and using prepared and packaged foods, due to financial problems and lack of time, were among the barriers of healthy eating in children (35, 70). As Lobstein et al. suggested, the governance and management of food supply and food markets need to be improved and commercial activities need to be increased to support and promote children's health (71).

Cultural beliefs on childhood obesity (56, 60, 66) were important barriers at the sociocultural level. Parents’ misconceptions of childhood obesity make them reluctant to use obesity preventive services in the healthcare system (35, 56). Studies show that a high percentage of parents with obese children and adolescents did not accept their children's obesity (72, 73). Therefore, it is necessary to construct cultural capacity-building to improve health literacy among children, adolescents, and parents and it is recommended that policymakers put COP initiatives as a political priority (60).

In this study, the relationship between stakeholders (58, 64, 67), parents, and school staff (54, 57) are the important facilitators of the sociocultural level. Effective communication is vital and critical to identify and address the stakeholders demands and needs (74). The impact of strengthening partnerships of stakeholders, especially the collaboration between healthcare providers as well as between healthcare providers and service recipients, has been well illustrated in the studies (58, 64, 67, 75, 76). Ciccone et al. (76) showed that the partnerships in the healthcare system lead to improved patient health knowledge and self-management skills, including self-management education and follow-up, as important components of the participatory approach (77). Adhikari et al. highlighted that trusted relationships among the key stakeholders are needed for the effective functioning of a health system (78). Consistent with the findings of the previously published scoping review (38), this review identified that factors related to environmental context, resources, and social influences had the most important impact on the policies related to this area such as physical activity policies.

The important barriers at the structural level in this review were limited funding and resources (47, 55, 61, 63–67), lack of support by experts (53, 57, 63, 65–67), and stakeholders’ time limitations in the implementation level (49, 51, 52, 60, 62, 66), which were similar to the results in the studies by Skea et al. (79) and Grady et al. (80). Similar to the present study, Heller et al. demonstrated that insufficient investment in the care delivery system is one of the key barriers in the delivery of care for noncommunicable diseases (81). Time limitations can be due to the low workforce and high workload at the executive level (60, 66). The studies indicated that the poor provision of school meals and the ease of access to cheap fast foods (33) have negative effects on healthy eating. Various interventions have been carried out to deal with the financial barriers in the low-income communities. For example, Dickin et al. showed that in the low-income communities, the policy of preventing childhood obesity was facilitated by increasing physical activity, introducing nutrition education in curricula, and hands-on workshops for parents (82, 83).

McPherson et al. suggested that policies should not only focus on the policy development stage but also encompass sufficient support for the optimal implementation of these policies; otherwise, these politics will not be successful (84). Nathan et al., in a systematic review study of the barriers and facilitators of the physical activity policies implementation in schools, demonstrated that program support is one of the most important factors of goal achievement in schools (38). For example, school-based COP policies can be supported by dealing with barriers, such as the lack of infrastructure near schools (51), obesogenic environments (54), junk food advertisement (56), and limited local control over food provided in schools (61).

At the structural level, the interventions with low cost, flexible and available features (49, 51, 56–58, 65), and delivery of healthy food in schools (51, 56), and appropriate support of intervention (58, 65) were considered as important and frequently reported facilitators. Some of the dimensions of these facilitators were in agreement of the previous review studies (68, 80, 85, 86). The reason why other facilitators were not examined in the study by Ray et al. could be because their study was only related to the opinions of the primary care providers toward practice behaviors and their perceptions of facilitators to implementing COP. In addition, the data related to the barriers and facilitators of the study by Ray et al. were attributions that primary care providers make about their own behaviors, not the actual determinants of their practices (68). The environment that was investigated in the study by Shoesmith et al. (85) was only schools and childcare services, and in Grady et al. (80) it was family day care setting; therefore, limiting their study environment led to the limited results. Many studies are needed to examine the gaps in this specific area, such as studies on the psychosocial stressors or exclusive breastfeeding and genetic (87).

## Conclusion

There is consistent qualitative evidence that several barriers and facilitators at various levels (e.g., individual, sociocultural, and structural) influence the implementation of COP policies. The policies may be well written in the policymaking stage, but they do not show good results due to not managing the barriers of their implementation or improper use of the facilitation. These findings support the rationale for the policymaking and development of multilevel interventions to reduce obesity in children and adolescents. The barriers to COP policy implementation have been studied more comprehensively than the facilitators. The diagnosis of numerous barriers and facilitators suggests that comprehensive strategies targeting these factors, especially examining the facilitators, to support the implementation of policies, may be required.

### Practice implications

Considering the implementation of COP policies and policies in practice, we face many barriers and problems with implementation; therefore, focusing on the barriers and facilitators, especially at the structural level, can help policymakers considering the barriers and facilitators identified in this study to address the long-term health outcomes in children.

## Data Availability

The raw data supporting the conclusions of this article will be made available by the authors, without undue reservation.
